# Lost in the Digital Void: The Interplay of Nomophobia, Loneliness, and Self-Esteem Among Medical Undergraduates of Central India

**DOI:** 10.7759/cureus.80087

**Published:** 2025-03-05

**Authors:** Neethu Baby, Sarita K Sharma, Pragati G Rathod, Ujwala U Ukey, Jay Prakash Gupta, Uday Narlawar, Kumari Rajnita, Deepika Nair, Anjali Vamadevan

**Affiliations:** 1 Community Medicine, Government Medical College and Hospital, Nagpur, IND

**Keywords:** loneliness, medical students, nomophobia, self-esteem, undergraduate

## Abstract

Introduction and aim: Nomophobia, also known as “no mobile phone phobia,” represents a mental condition caused by the fear of being detached from mobile phone connectivity. Loneliness and self-esteem are two psychological factors often associated with nomophobia. This study aimed to identify the pattern of mobile use to explore the prevalence of nomophobia, loneliness, and self-esteem among undergraduate medical students of Central India. It also aimed to assess the relationship of nomophobia with loneliness and self-esteem among them.

Methods: A cross-sectional study was conducted among 316 undergraduate medical students of Government Medical College, Nagpur from August 2023 to October 2023. Data were collected using a predesigned, pretested, and standardized questionnaire. Nomophobia was assessed using Nomophobia Scale, loneliness by using the University of California, Los Angeles (UCLA) Loneliness Scale, and self-esteem was assessed using the Rosenberg Self-Esteem Scale. Karl Pearson correlation coefficient (r) was used to correlate the scores.

Results: There were 162 (51.3%) females and 154 (48.7%) males and the mean age was 21±1.72 years. More than 50% of the students had mild-to-moderate levels of nomophobia. The majority of the students had moderate levels of loneliness and self-esteem. There was a significant positive correlation between nomophobia and level of loneliness (r=0.99). The study found that 35.75% of participants exhibited low self-esteem. A statistically significant negative correlation (r=-0.32, p=0.05) was observed between nomophobia and self-esteem.

Conclusion: The high prevalence of nomophobia highlights the extent of mobile phone dependency in this population. A significant positive correlation was found between nomophobia and loneliness, suggesting that excessive reliance on mobile phones might be linked to a lack of meaningful social interactions or heightened feelings of isolation.

## Introduction

Advances in information and communication technologies have made smartphones essential to modern life, providing services that extend far beyond basic communication. As these devices become increasingly affordable and indispensable, mobile dependency has surged globally [1-3]. These devices offer a range of services beyond calling and texting, such as emailing, scheduling appointments, browsing the internet, shopping, social networking, searching for information, gaming, and more [4]. However, in high-pressure academic settings such as medical colleges-this dependency may have adverse effects on mental well-being [5,6].

The term nomophobia, also known as “no mobile phone phobia,” was first coined during a study conducted in 2008 by the UK Post Office to investigate anxieties mobile phone users suffer. This condition has gained significant attention with the increasing reliance on smartphones for communications, entertainment, and social connections. Nomophobia, the fear of being out of mobile phone contact, can trigger anxiety when individuals experience no network, low battery, or insufficient balance. This anxiety may, in turn, reduce their ability to concentrate [7-9].

Two key psychological factors - loneliness and self-esteem - are closely linked to nomophobia. Loneliness, defined as the perceived absence of meaningful social connections, may drive individuals to seek solace in their mobile devices, while excessive phone use can, in turn, intensify feelings of isolation [10]. Self-esteem refers to an individual's overall subjective evaluation of their worth and confidence in their abilities [11]. Low self-esteem may lead to increased mobile phone reliance as a coping mechanism, further reinforcing nomophobic behaviors. These factors share a bidirectional relationship as follows: chronic loneliness can erode self-worth, while diminished self-esteem may hinder the formation of social connections, further deepening feelings of isolation [12].

Nomophobia thus is a growing concern globally, with studies indicating its association with increased anxiety, loneliness, and lower self-esteem. However, there is limited research on its impact specifically among undergraduate medical students in India. This study aimed to bridge that gap by analyzing the correlation between nomophobia and psychological factors among this group. The healthcare industry can leverage this knowledge to develop targeted interventions and counseling, to mitigate the negative effects of excessive smartphone use.

## Materials and methods

Study design, setting, and duration

This was a cross-sectional study conducted to assess nomophobia and its associations with loneliness and self-esteem among undergraduate medical students. The study was carried out at Government Medical College, Nagpur, Maharashtra, a well-established teaching institution with an annual intake of 250 undergraduate students. Data collection took place over a period of three months, from August 2023 to October 2023, using an online self-administered questionnaire.

Sample size calculation

The required sample size was determined based on the prevalence of nomophobia reported in a previous study by Sethia et al. which documented a 67% prevalence rate [12]. Considering a 95% confidence interval, a 10% allowable error, and an additional 10% non-response rate, the final estimated sample size was 316 students.

Study population

The study recruited 316 undergraduate medical students who met the inclusion criteria. Participants were selected using a convenience sampling technique from the first, second, and final-year MBBS cohorts. The inclusion criteria cover current smartphone users enrolled in these academic years, regardless of gender. Students with a history of psychiatric disorders such as anxiety, or depression, as well as those undergoing current psychiatric treatment, were excluded. Additionally, students who did not provide informed written consent were not included in the study.

Data collection tools

The data collection instrument was a pretested and validated self-administered structured questionnaire comprising three sections: part A collected general demographic information such as age, gender, marital status, and year of study, as well as details of mobile phone usage patterns. Part B employed the Nomophobia Questionnaire (NMP-Q) to assess the severity of nomophobia [2]. The Nomophobia Questionnaire (NMP-Q) consists of 20 items, categorized into four dimensions - losing connectivity, inability to communicate, lack of access to information, and smartphone-related anxiety. Part C incorporated the University of California, Los Angeles (UCLA) Loneliness Scale [8] and Rosenberg Self-Esteem Scale to evaluate loneliness and self-esteem, respectively [11]. The University of California, Los Angeles (UCLA) Loneliness Scale is a 20-item tool measuring subjective feelings of loneliness and social isolation whereas the Rosenberg Self-Esteem Scale is a 10-item self-report questionnaire evaluating self-esteem. The reliability of the instruments was confirmed with acceptable Cronbach’s alpha coefficients - Nomophobia Questionnaire (NMP-Q: 0.91), UCLA Loneliness Scale (0.89), and Rosenberg Self-Esteem Scale (0.85). All identifiable participant data were de-identified to maintain confidentiality. Data were stored securely, and access was restricted to authorized researchers only.

Nomophobia Questionnaire (NMP-Q) was rated on a seven-point Likert scale. Total scores range from 20 to 140, categorized as mild (20-59), moderate (60-99), and severe (100-140) nomophobia [2]. University of California, Los Angeles (UCLA) Loneliness Scale was scored on a four-point Likert scale. Total scores range from 20 to 80. The scores between 20 and 34 indicate low loneliness, 35 and 49 suggest moderate loneliness, 50 and 64 represent high loneliness, and scores 65 and above indicate severe loneliness [8]. The Rosenberg Self-Esteem Scale (RSES) is a widely used psychological tool designed to measure an individual's overall self-esteem. This scale consists of 10 items, rated on a four-point Likert scale as follows: strongly disagree (1), disagree (2), agree (3), and strongly agree (4). Five of the items (2, 5, 6, 8, and 9) are negatively worded (e.g., "At times I think I am no good at all") and are reverse-scored before calculating the total score. The total score ranges from 10 to 40, with higher scores reflecting higher self-esteem. A score of 30-40 is generally interpreted as high self-esteem, 20-29 as moderate self-esteem, and 10-19 as low self-esteem [11].

Statistical analysis

Data analysis was performed using SPSS (trial version 29; Armonk, NY: IBM Corp.). Descriptive statistics, including frequencies and proportions, were used to summarize the data. The chi-square test was applied to examine the relationship between the severity of nomophobia and different smartphone usage patterns. A p-value of <0.05 was considered statistically significant. Additionally, the Karl Pearson correlation coefficient (r) was employed to determine the associations between nomophobia scores and measures of loneliness and self-esteem among the students.

## Results

Out of 316 students included in the study, 154 (48.7%) were males and 162 (51.3%) were females, the mean age was 21±1.72 years. Table 1 shows demographic profiles of the study participants. A striking 98.73% of participants exhibited nomophobia. Among them, 198 (63%) had moderate nomophobia, 62 (20%) had severe, and 52 (17%) reported mild nomophobia (Figure 1).

**Table 1:** Demographic profiles of the study participants. N=total number

Variables	Number (N=316)	Percentage
Age (years)		
18-21	211	66.8
22-25	105	33.2
Gender		
Males	154	48.7
Females	162	51.3
Year of study		
First year	62	19.6
Second year	42	13.3
Third year	195	61.7
Fourth year	17	5.4

**Figure 1:** Severity levels of nomophobia.

The relationship between the severity of nomophobia and the pattern of smartphone use is presented in Table 2. The severity of nomophobia demonstrated a significant association with the duration of smartphone use per day (p=0.006). The frequency of smartphone checking exhibited a statistically significant association with the severity of nomophobia (p=0.046). An increased number of applications on the phone was also linked to heightened nomophobia severity, with a statistically significant association (p=0.013).

**Table 2:** Relationship between severity of nomophobia and pattern of smart phone use. *The values were calculated using chi-square test. **P<0.05 was considered statistically significant.

Pattern of smartphone use		Nomophobia		p-Value*
		Moderate-to-severe (%)	Mild (%)	
Duration of smartphone use (years)	Less than 2	21 (67.74)	8 (25.8)	0.253
	2-5	162 (83.93)	30 (15.54)	
	More than 5	77 (83.7)	14 (15.21)	
Duration of smartphone use (hours) in a day	Less than 2	13 (65)	5 (25)	0.006**
	2-5	115 (68.45)	52 (30.95)	
	More than 5	108 (84.37)	19 (14.84)	
Having mobile data plan	Yes	255 (82.52)	50 (16.18)	0.330
	No	5 (71.42)	2 (28.57)	
Frequency of checking smartphone	Once every half an hour	99 (86.84)	12 (10.52)	0.046**
	Once every half an hour to an hour	110 (82.70)	23 (17.29)	
	Once beyond an hour	51 (73.91)	17 (24.63)	
Number of applications in the phone	Less than 20	79 (74.52)	24 (22.64)	0.013**
	20-50	140 (84.33)	25 (15.06)	
	More than 50	42 (95.45)	2 (4.54)	

Figure 2 illustrates the levels of loneliness among the study participants, categorized into low, moderate, and high. The majority 228 (72%) experienced moderate loneliness, while 57 (18%) reported low loneliness, and 31 (10%) had high levels of loneliness.

**Figure 2:** Levels of loneliness.

Nomophobia displayed a positive correlation with loneliness (r=0.99), although this correlation was not found to be statistically significant (p=0.06) (Figure 3). Figure 4 depicts the levels of self-esteem among the study participants, categorized as low, moderate, and high. The majority 135 (43%) had moderate self-esteem, followed by 113 (36%) with low self-esteem, while only 68 (21%) reported high self-esteem.

**Figure 3:** Scatter diagram showing the correlation between nomophobia and loneliness. Here, y represents the predicted values of self-esteem, while R² denotes the coefficient of determination, indicating the strength of the relationship between nomophobia and self-esteem.

**Figure 4:** Levels of self-esteem.

It was observed that nomophobia exhibited a statistically significant negative correlation with self-esteem (r=-0.32), emphasizing the interplay between these factors (p=0.05) (Figure 5). The study's results indicate a high prevalence of nomophobia among undergraduate medical students, with notable associations between nomophobia severity, smartphone use patterns, and psychosocial aspects such as loneliness and self-esteem.

**Figure 5:** Scatter diagram showing the correlation between nomophobia and self-esteem. Here, y represents the predicted values of self-esteem, while R² denotes the coefficient of determination, indicating the strength of the relationship between nomophobia and self-esteem.

## Discussion

Smartphones have emerged as an example of “a paradox of technology,” with both the property of freeing and enslaving [7]. Freeing from the real world and enslaving to the virtual world [7]. The current study highlights the pervasive issue of nomophobia (the fear of being without a mobile phone) among medical undergraduates with four-fifths of them exhibiting moderate-to-severe nomophobia. These results align with those of previous research conducted in a medical college in Kerala, where the prevalence of nomophobia was reported to be 97% [10]. Similarly, Sethia et al. observed that nearly every participant in their study experienced some level of nomophobia, with 6.1% reporting severe nomophobia [12].

Cain and Malcom reported an overwhelming prevalence of 99.5% among students in the United States [13], while research conducted in Oman indicated a similar rate of 99.33% [14]. A recent study from Saudi Arabia documented an 85.3% prevalence of nomophobia among university students [15]. The high incidence of nomophobia among medical students is a growing concern that demands greater awareness and intervention. Given the academic pressures and demanding nature of medical education, students heavily depend on their smartphones, making them particularly susceptible to this condition.

Conversely, two Indian studies reported significantly lower prevalence rates. One study found that only 25.21% of students experienced nomophobia [16], whereas another study revealed that 50.70% had moderate nomophobia, while 30.26% suffered from severe forms of the condition [17]. Variations in study populations, assessment tools, and methodologies may contribute to the discrepancies observed in prevalence rates across different studies. It is concerning that the proportion of individuals with severe nomophobia appears to be increasing, particularly among medical students because this could have significant implications for their well-being and academic performance.

In terms of pattern of smartphone usage, most participants reported using their devices more than 5 hours a day. This pattern of usage is consistent with the findings of Chethana et al. who similarly observed that students frequently used smartphones for longer duration in a day [18]. In this context, the findings of this study also align with previous research conducted in Saudi Arabia, where most participants reported spending more time online than they initially expected [19]. The ubiquitous presence of smartphones and their multifunctional capabilities make them indispensable in the daily lives of students, further contributing to the dependence that characterizes nomophobia.

A notable finding from the current study is the positive correlation between nomophobia and perceived loneliness, coupled with a negative correlation between nomophobia and self-esteem. Nomophobia and loneliness are interconnected; reliance on smartphones to alleviate loneliness often fosters superficial digital interactions, deepening isolation. This dependence creates a feedback loop, reducing face-to-face connections and exacerbating social withdrawal, thus leading to loneliness. The statistically significant association between nomophobia and low self-esteem mirrors the results reported by Ozdemir et al. Nomophobia and low self-esteem are closely linked, as individuals with low self-esteem often rely on mobile phones for external validation, social connection, and escapism. This dependence reinforces anxiety when phones are unavailable, exacerbating feelings of inadequacy and fear of exclusion [19,20].

Additionally, the study by Çakir and Oguz in 2017, conducted among Turkish students, demonstrated a similar relationship between smartphone addiction and loneliness [21]. This correlation between smartphone dependence and loneliness has been echoed in other studies, including one conducted among Japanese medical students, which found that increased mobile phone dependence was linked to higher levels of loneliness and addiction [22]. These findings are consistent with a study conducted in Turkey, which identified a strong positive relationship between nomophobia and loneliness [23]. Similarly, research by Kayis et al. on the Turkish general population found a moderate yet significant correlation between loneliness and smartphone dependency [24].

These findings suggest that the growing reliance on smartphones is not only altering social behaviors but may also contribute to mental health issues such as anxiety, loneliness, and depression [25-28]. Strengths of the present study include the use of validated scales, a relatively large sample size, and a focus on an at-risk population. However, the present study has some limitations like those related to the cross-sectional design, potential response bias, and limited generalizability because the data were collected from a single institute. While limitations exist, this study provides valuable insights into nomophobia's psychological effects on medical students. Addressing these issues early can help in framing policies on mental health and digital well-being for medical students.

## Conclusions

The increasing prevalence of nomophobia, particularly among medical students, is a matter of growing concern. With a sizeable proportion of participants in the present study suffering from severe nomophobia, and nomophobia exhibiting a strong correlation with both loneliness and self-esteem, the findings highlight the negative psychological impacts of excessive smartphone use. The rising dependence on mobile phones may have long-term consequences, leading to mental health challenges, and underscores the importance of addressing this issue within the context of student health and well-being. Initiatives like awareness campaigns, mental health counseling, and digital detox can help students reduce their reliance on their devices.

By addressing nomophobia early and promoting balanced smartphone use, institutions can help mitigate its adverse effects and support the overall mental health of students. Further, longitudinal studies are needed to explore the long-term effects of nomophobia on the mental health and academic performance of students. Also, future research can cover topics like apps/applications used by the students and their effect on their mental health.
